The article "Efficacy Evaluation of High-Volume Hemofiltration in Patients with Severe Acute Respiratory Distress Syndrome" was retracted in 2023. Reasons: signs of a paper mill; suspected computer-generated content; unreliable results or conclusions; concerns about the data.

# Efficacy Evaluation of High-Volume Hemofiltration in Patients with Severe Acute Respiratory Distress Syndrome

**DOI:** 10.1155/2022/9488047

**Published:** 2022-09-20

**Authors:** Yonglei Zhang, Yan Zhang, Jiming Pan

**Affiliations:** Department of Emergency Intensive Care, Yantaishan Hospital, Yantai, China

## Abstract

**Objective:**

To investigate the efficacy of high-volume hemofiltration (HVHF) in the treatment of severe acute respiratory distress syndrome (ARDS) caused by sepsis and its effect on serum levels of miR-126, miR-184, and MAP1-LC3.

**Methods:**

From July 1, 2015 to December 31, 2021, patients with severe ARDS caused by sepsis who were admitted to our hospital were retrospectively analyzed. Patients who received conventional treatment were summarized into the control group, and those who received HVHF were summarized into the study group. The treatment effects of the two groups were compared.

**Results:**

Ninety-five qualified patients were retrieved, with 42 patients in the control group and 53 patients in the study group. After treatment, the levels of IL-6, IL-10, TNF-*α*, miR-126, miR-184, and MAP1-LC3 were significantly lower in the study group (*P* < 0.05 for all), whereas PEF, FRC, TEF25%, heart rate, mean arterial pressure, and blood oxygen were significantly higher in the study group (*P* < 0.05 for all).

**Conclusion:**

HVHF has a good clinical effect on improving patients with severe ARDS caused by sepsis and can improve the pulmonary function of patients.

## 1. Introduction

Sepsis, a systemic inflammatory response syndrome (SIRS) caused by infection, is characterized by a high mortality rate and is commonly seen in intensive care units [1, 2]. The pathogenesis of acute respiratory distress syndrome (ARDS) is caused by acute events, which can cause damage to the capillaries and epithelial cells in the lung, thereby causing diffuse edema of the lung tissue that leads to acute hypoxic respiratory failure. In recent years, anti-infection and multiorgan support technologies have made great progress, but the mortality rate of sepsis is still high [3]. High-volume hemofiltration (HVHF) technology has been shown to remove inflammatory mediators in blood purification technology, enhance antigen presentation, leukocyte activity, and body immunity, and can significantly improve lung function and blood oxygen concentration in ARDS patients [4]. This study aims to investigate the clinical effect of continuous HVHF in patients with severe ARDS.

## 2. Materials and Methods

### 2.1. General Information

From July 1, 2015 to December 31, 2021, patients with severe ARDS caused by sepsis who were treated in our hospital were retrospectively analyzed. All patients in this study signed the informed consent form. This study was approved by the Institutional Ethical Committee of our hospital.

Inclusion criteria were as follows: the clinical diagnosis was severe ARDS caused by sepsis [3]; severe hypoxia PaO_2_/Fi O_2_ ≤ 100 mm·Hg; PEEP ≥ 5 cm H_2_O; onset time ≤ 72 h, and oxygenation index ≤ 100 [5].

Exclusion criteria were as follows: complicated with malignant diseases, mental illness, drug allergies, etc.; patients aged ≤18 years or ≥75 years old; patients with liver or renal insufficiency; or patients with previous pulmonary underlying diseases.

### 2.2. Methods

Patients in the conventional treatment received mechanical ventilation, anti-infection, moderate fluid replacement, antishock, nutritional support treatment, etc. Patients in the research group received continuous HVHF on the basis of conventional treatment. The vascular access was established through the femoral vein, the replacement fluid was bicarbonate, the replacement fluid was diluted 80% before use, the flow rate of hemofiltration was 45 ml/kg/h, and heparin was used for anticoagulation. Continuous HVHF treatment was carried out for 24 hours, at least 3 days.

### 2.3. Observation Indicators

The inflammatory cytokines, lung function, serum miR-126, miR-184, MAP1-LC3 as previously reported [6], heart rate, mean arterial pressure, and blood oxygen were compared between the two groups.

### 2.4. Statistical Methods

The data in this experiment were analyzed by the SPSS21.0 software package (IBM Corp., Armonk, N.Y., USA), in which the count data were analyzed by *χ*^2^ test (*n*, %), and the measurement data were analyzed by *t*-test (mean ± SD). A two-tailed *P* < 0.05 was determined to have statistical significance.

## 3. Results

### 3.1. General Conditions of Enrolled Patients

There were 95 qualified patients retrieved. There was no difference in age, gender, or oxygenation index between the two groups (Table 1).

### 3.2. Comparison of Serum Cytokines between the Two Groups before and after Treatment

Before treatment, the levels of IL-6 (35.41 ± 5.26), IL-10 (48.62 ± 7.33), and TNF-*α* (9.15 ± 1.22) in the study group were comparable with the control group IL-6 (35.27 ± 5.35), IL-10 (48.37 ± 7.25), and TNF-*α* (9.13 ± 1.25), without significant difference (*F* = 3.330, 2.025, 2.551, *P*=0.051, 0.301, 0.210). After treatment, IL-6 (9.25 ± 1.38), IL-10 (16.29 ± 2.64), and TNF-*α* (3.17 ± 0.45) were significantly lower than the control group IL-6 (21.38 ± 3.42), IL-10 (34.52 ± 5.58), and TNF-*α* (5.58 ± 0.82). See Table 2 for details.

### 3.3. Serum Levels of MiR-126, MiR-184, and MAP1-LC3 in the Two Groups

Before treatment, the miR-126 (2.06 ± 0.23), miR-184 (12.64 ± 4.17), and MAP1-LC3 (1.07 ± 0.01) of the study group were comparable with the control group of miR-126 (2.05 ± 0.06), miR-184 (12.07 ± 4.24), and MAP1-LC3 (1.05 ± 0.38), and the differences were not statistically significant (*P* > 0.05). However, the levels of miR-126, miR-184, and MAP1-LC3 in the two groups after treatment were both significantly lower than those before the treatment, and the levels of miR-126, miR-184, and MAP1-LC3 were significantly lower in the study group than those in the control group (Table 3).

### 3.4. Comparison of Lung Function between the Two Groups before and after Treatment

Before treatment, the study group had comparable PEF (46.35 ± 7.29), FRC (64.88 ± 8.48), and TEF25% (42.07 ± 4.83) as the control group PEF (42.07 ± 4.83), FRC (65.27 ± 8.33), and TEF25% (41.44 ± 5.27), and there were no significant differences (*P* > 0.05). After treatment, the PEF (67.10 ± 7.28), FRC (90.74 ± 8.63), and TEF25% (54.28 ± 5.27) of the study group were significantly higher than the control group PEF (60.17 ± 8.07), FRC (84.45 ± 9.46), and TEF25% (49.85 ± 5.12) (*F* = 3.54, 6.35, 6.16, *P* < 0.05, Table 4).

### 3.5. Comparison of Heart Rate, Mean Arterial Pressure, and Blood Oxygen between Two Groups of Patients

Before treatment, the heart rate (64.10 ± 1.22), mean arterial pressure (80.15 ± 5.42), and blood oxygen (95.15 ± 2.33) of the study group were comparable with the control group heart rate (63.25 ± 1.03), mean arterial pressure (80.23 ± 2.35), and blood oxygen (94.10 ± 2.53), with no significant differences (*P* > 0.05). After treatment, the heart rate (82.73 ± 2.54), mean arterial pressure (92.45 ± 0.27), and blood oxygen (98.10 ± 1.01) of the study group were significantly higher than the control group heart rate (65.58 ± 2.67), mean arterial pressure (81.53 ± 1.85), and blood oxygen (95.10 ± 1.20) (*F* = 4.91, 4.11, 5.89, *P* < 0.05, Table 5).

## 4. Discussion

Sepsis, an unusual systemic response to common infection or intestinal ischemia/reperfusion, may represent a pattern in the immune system's response to injury [7]. An excessive inflammatory response is followed by a phase of immunosuppression, during which multiple organ dysfunction is present and the patient is susceptible to nosocomial infections. ARDS is a nonhydrostatic pulmonary edema and hypoxemic process associated with multiple etiologies with high morbidity and mortality (10% to 90%) characterized by increased permeability of the alveolar-capillary barrier, resulting in alveolar leukocyte infiltration and protein-rich pulmonary edema [8]. The clinical presentation was refractory hypoxemia and bilateral pulmonary infiltrates, with no evidence of left heart failure or volume overload [9]. ARDS is primarily driven by inflammatory chemokines and cytokines that are endogenously produced in response to various stimuli and events [10]. In children, one study reported a mortality rate of approximately 10% for mild and moderate ARDS and as high as 25% for severe ARDS. Inhaled oxygen (PaO_2_/FiO_2_) is closely related to mortality [11]. Hemofiltration has been proposed as a possible therapeutic option to improve oxygenation by promoting fluid removal, but its efficacy remains controversial. Several studies have concluded that continuous renal replacement therapy (CRRT), indicated for acute fluid overload (FO) and acute renal failure, improves oxygenation in patients with respiratory failure, hypoxia, and fulminant hepatitis [12–18]. However, others found no improvement in oxygenation. Even though CRRT can improve oxygenation in ARDS patients, it remains controversial whether the beneficial effects on pulmonary gas exchange are mediated by mechanisms other than fluid removal, such as through sustained removal of inflammatory mediators. miR-126, miR-184, and MAP1-LC3 have been used as markers for ARDS [6], which were employed in this study to show the efficacy of HVHF.

Extracorporeal blood purification is often used to deal with poisoning. Hemofiltration removes solutes from plasma through a membrane induced by a pressure gradient [12]. HVHF is defined as continuous high-volume treatment with an ultrafiltration rate exceeding 50 mL/kg/ha per day. There are many different hypotheses about how HVHF attenuates the overexpression of systemic inflammatory mediators, restores immune homeostasis, and ultimately improves clinical outcomes. Although HVHF is frequently used for acute kidney injury, extensive experimental and some clinical evidence suggests that HVHF is effective in reducing the levels of precursors and anti-inflammatory mediators associated with systemic inflammatory response syndrome (SIRS) and multiple organ dysfunction syndrome (MODS), which are beneficial in critically ill patients with severe inflammatory states [12]. It has the functions of expelling excess water in the human body, regulating the acid-base balance, and reducing the damage to lung tissue caused by pulmonary edema and hypercapnia; it also clears inflammatory mediators and toxin molecules and has a certain impact on the body's immune function. HVHF also improves hemodynamics, reduces myocardial damage, and prevents the occurrence of disseminated intravascular coagulation (DIC) and immune paralysis.

Continuous HVHF can meet the treatment needs of sepsis, but due to the different metabolic and infectious conditions of patients, there is no uniform rate standard. However, it is certain that it is very effective in the treatment of sepsis. In the process of HVHF, the rate of replacement fluid has a great relationship with the removal rate. Early and accurate diagnosis of ARDS would lead to a therapeutic advantage, and the findings of our study will provide valuable clues for the application of traditional Chinese medicine.

In conclusion, HVHF has a good clinical effect in improving patients with severe ARDS caused by sepsis and can improve the pulmonary function of patients.

## Figures and Tables

**Table 1:** General information of patients.

Generally	Study group	Control group	*t*/*χ*^2^	*P*
*N*	53	42		

Age	58.51 ± 3.36	57.96 ± 4.02	0.7263	0.470

Gender			0.255	0.614
Male	28	20		
Female	25	22		

Oxygenation index	80.28 ± 4.27	79.35 ± 5.14	0.9632	0.338

**Table 2:** Serum cytokine levels in two groups of children (pg/ml, $\bar{x}\pm s$).

Group	Control group (*n* = 42)	Study group (*n* = 53)	Ft/Fg	Pt/Pg
IL-6				
Before therapy	35.27 ± 5.35	35.41 ± 5.26	3.330/8.450	0.051/0.004
After treatment	21.38 ± 3.42^	9.25 ± 1.38^^*∗*^		

IL-10				
Before therapy	48.37 ± 7.25	48.62 ± 7.33	2.025/6.171	0.301/0.001
After treatment	34.52 ± 5.58^	16.29 ± 2.64^^*∗*^		

TNF-*α*				
Before therapy	9.13 ± 1.25	9.15 ± 1.22	2.551/9.551	0.210/0.003
After treatment	5.58 ± 0.82^	3.17 ± 0.45^^*∗*^		

Note: Ft and Pt are the statistical values of time; Fg and Pg are the statistical values of factors between groups; compared with the control group, ^*∗*^*P* < 0.05; compared with before treatment, ^*P* < 0.05.

**Table 3:** Serum levels of miR-126, miR-184, and MAP1-LC3 in the two groups.

Group	Control group (*n* = 42)	Study group (*n* = 53)	Ft/Fg	Pt/Pg
miR-126				
Before therapy	2.05 ± 0.06	2.06 ± 0.23	5.08/4.14	0.02/0.04
After treatment	1.06 ± 0.13^	0.94 ± 0.52^^*∗*^		

miR-184				
Before therapy	12.07 ± 4.24	12.64 ± 4.17	4.59/6.20	0.03/0.01
After treatment	5.18 ± 1.33^	2.25 ± 1.61^^*∗*^		

MAP1-LC3				
Before therapy	1.05 ± 0.38	1.07 ± 0.01	4.31/6.78	0.04/0.01
After treatment	0.60 ± 0.17^	0.41 ± 0.12^^*∗*^		

Note: Ft and Pt are the statistical values of time; Fg and Pg are the statistical values of factors between groups; compared with the control group, ^*∗*^*P* < 0.05; compared with before treatment, ^*P* < 0.05.

**Table 4:** Pulmonary function of the two groups of patients.

Group	Control group (*n* = 42)	Study group (*n* = 53)	F_t_/F_g_	P_t_/P_g_
PEF (ml/s)				
Before therapy	45.86 ± 7.91	46.35 ± 7.29	4.12/3.54	0.01/0.02
After treatment	60.17 ± 8.07^	67.10 ± 7.28^^*∗*^		

FRC (ml)				
Before therapy	65.27 ± 8.33	64.88 ± 8.48	4.37/6.35	0.02/0.01
After treatment	84.45 ± 9.46^	90.74 ± 8.63^^*∗*^		

TEF25% (ml)				
Before therapy	41.44 ± 5.27	42.07 ± 4.83	4.26/6.16	0.03/0.01
After treatment	49.85 ± 5.12^	54.28 ± 5.27^^*∗*^		

Note: Ft and Pt are the statistical values of time; Fg and Pg are the statistical values of factors between groups; compared with the control group, ^*∗*^*P* < 0.05; compared with before treatment, ^*P* < 0.05.

**Table 5:** Comparison of heart rate, mean arterial pressure, and blood oxygen in the two groups of patients.

Group	Control group (*n* = 42)	Study group (*n* = 53)	Ft/Fg	Pt/Pg
Heart rate (beats/min)				
Before therapy	63.25 ± 1.03	64.10 ± 1.22	5.00/4.91	0.03/0.03
After treatment	65.58 ± 2.67^	82.73 ± 2.54^^*∗*^		

Mean arterial pressure (mmHg)				
Before therapy	80.23 ± 2.35	80.15 ± 5.42	6.26/4.11	0.01/0.04
After treatment	81.53 ± 1.85^	92.45 ± 0.27^^*∗*^		

Blood oxygen				
Before therapy	94.10 ± 2.53	95.15 ± 2.33	4.54/5.89	0.03/0.02
After treatment	95.10 ± 1.20^	98.10 ± 1.01^^*∗*^		

## Data Availability

Data will be made available from the corresponding author upon request.
